The article "Low Serum Albumin Is Associated with Poor Prognosis in Patients Receiving Peritoneal Dialysis Treatment" was retracted in 2023. Reasons: signs of a paper mill; suspected computer-generated content; unreliable results or conclusions; concerns about the data.

# Low Serum Albumin Is Associated with Poor Prognosis in Patients Receiving Peritoneal Dialysis Treatment

**DOI:** 10.1155/2022/7660806

**Published:** 2022-04-18

**Authors:** Yanan Shi, Jiajie Cai, Chunxia Shi, Conghui Liu, Jingjing Zhou, Zhongxin Li

**Affiliations:** Department of Nephrology, Beijing Lu-He Hospital, Capital Medical University, Beijing 101100, China

## Abstract

**Background:**

The number of patients receiving dialysis treatment is sustainably increasing, especially peritoneal dialysis.

**Objectives:**

It is necessary to find out potential factors that may indicate the prognosis of patients receiving peritoneal dialysis treatment.

**Methods:**

This study retrospectively involved 325 patients who received peritoneal dialysis treatment.

**Results:**

Low serum albumin (HR = 2.254; 95% CI: 1.534–3.311; *P* < 0.001) and high FBG (Fasting blood glucose) (HR = 1.474; 95% CI: 1.025–2.120; *P*=0.037) were risk factors for death in patients receiving peritoneal dialysis treatment. Serum albumin (AUC = 0.683; *P* < 0.001) and creatinine (AUC = 0.625; *P* < 0.001) exhibited value of prognosis prediction. Both high FBG (*P*=0.005) and low albumin (*P* < 0.001) were associated with poor prognosis, and low albumin predicted poorer survival.

**Conclusions:**

Low serum albumin and high fasting blood glucose were risk factors and associated with poor prognosis. Low albumin has a potential in predicting the prognosis of patients receiving peritoneal dialysis treatment.

## 1. Introduction

Dialysis is a renal replacement therapy (RRT), mainly including hemodialysis and peritoneal dialysis [1, 2]. The principle of peritoneal dialysis is the solutes and fluid exchange between the peritoneal capillary blood and the dialysis solution, in which the flow rate can be adjusted to achieve a maximum removal [2]. It is estimated that more than 272,000 patients are receiving peritoneal dialysis globally, accounting for approximately 11% dialysis patients worldwide (in 2017) [3]. The number of patients receiving dialysis treatment is sustainably increasing, especially peritoneal dialysis [4]. Among different countries, the selection of dialysis modality is dramatically different [3]. Different dialysis modalities bring important consequences for quality of life, patients' survival, financial implications, and logistics for the medical system [1, 5]. In Asia, the application of peritoneal dialysis ranges from 3% to 73%, and China has a fairly high peritoneal dialysis rate [3, 4, 6]. Notably, there is a steep rise in peritoneal dialysis utilization in China in the past decade [7].

Albumin is a single protein species and the most abundant plasma protein representing approximately 3/5 in quantity [8]. Albumin produced in the liver is an anionic, flexible, heart-shaped molecule with a molecular weight of ∼65 kDa [9]. Normally, the serum albumin is about 45 g/L in human. Albumin plays an important role in maintaining an oncotic pressure difference between plasma and the interstitial space by regulating fluid exchange [10]. Besides, albumin carries a number of substances including bilirubin, fatty acids, ions, hormones, and drugs [8, 10]. Notably, low albumin in serum is in association with increased mortality [10].

The article "Low Serum Albumin Is Associated with Poor Prognosis in Patients Receiving Peritoneal Dialysis Treatment" was retracted in 2023. Reasons: signs of a paper mill; suspected computer-generated content; unreliable results or conclusions; concerns about the data.

It is necessary to find out potential factors that may indicate the prognosis of patients receiving peritoneal dialysis treatment. Herein, factors associated with the prognosis of patients receiving peritoneal dialysis treatment, such as serum albumin, creatinine, and fasting blood glucose, were evaluated. We also compared their abilities of prognosis prediction by ROC (receiver operating characteristic) analysis and survival analysis.

## 2. Materials and Methods

### 2.1. Patients

This study retrospectively involved 325 patients who received peritoneal dialysis treatment. Each patient had a complete record of dialysis during the period. All lab parameters were measured at admission as a baseline. The follow-up duration was 7 years.

Patients who were older than 18 years old and received peritoneal dialysis treatment for more than 3 months were included.

The exclusion criteria were as follows: incubation in other hospitals, hemodialysis to peritoneal dialysis, kidney transplant to peritoneal dialysis, annual follow-up <2, and missing baseline data.

### 2.2. Clinical Data Collection

After admission, the age of patients was recorded, and systolic pressure, diastolic pressure, and pulse were measured. Moreover, the patients received laboratory examination including total protein (g/L), albumin (g/L), Ca^2+^ (mmol/L), phosphate (mmol/L), K^+^ (mmol/L), Na^+^ (mmol/L), Cl^−^ (mmol/L), fasting blood glucose (FBG; mmol/L), blood urea nitrogen (BUN; mmol/L), creatinine (*μ*moI/L), hemoglobin (g/L), and parathyroid hormone (PTH; pg/mL) test. Normal, low, and high individual parameters were defined according to the clinical standard of the clinical lab of our hospital.

### 2.3. Statistical Analysis

Software SPSS 22.0 (IBM, USA) was used. Data were exhibited as mean ± SD. Quantitative data are expressed as mean ± standard deviation or median (interquartile range). Qualitative data are expressed as a rate or composition ratio. Differences between groups were analyzed by the *T*-test or analysis of variance. Survival risk analysis was performed using a cox risk regression model. The ROC (receiver operating characteristic) curve was used to predict the risk of death for patients receiving peritoneal dialysis treatment, and the AUC (area under curve) was calculated. *P* < 0.05 was considered statistically significant.

The article "Low Serum Albumin Is Associated with Poor Prognosis in Patients Receiving Peritoneal Dialysis Treatment" was retracted in 2023. Reasons: signs of a paper mill; suspected computer-generated content; unreliable results or conclusions; concerns about the data.

## 3. Results

### 3.1. Characteristics of Patients Receiving Peritoneal Dialysis Treatment

The summary of all the characteristics of patients receiving peritoneal dialysis treatment is shown in Table 1. The average age was 62.51 years old. Among the 325 patients, 147 were male and 178 were female. The average survival time was 892.36 days.

### 3.2. Differences between Survived Patients and Dead Patients

The subsequent comparisons between the survival and the death were further performed (Table 2). No significant differences were found in gender (*P*=0.651), systolic pressure (*P*=0.198), pulse (*P*=0.745), total protein (*P*=0.092), Ca^2+^ (*P*=533), phosphate (*P*=0.467), K^+^ (*P*=0.322), Na^+^ (*P*=0.260), Cl^−^ (*P*=0.390), FBG (*P*=0.333), BUN (*P*=0.251), and PTH (*P*=0.882). Survival time (*P*=0.049) and diastolic pressure (*P*=0.047) showed a little statistical difference. The hemoglobin (*P*=0.038) was statistically different.

The age was significantly different (*P* < 0.001) as the dead patients (66.96 ± 13.89 years old) were much older than the survived patients (28.75 ± 13.13 years old).

The albumin was significantly different (*P* < 0.001) as the albumin in dead patients (32.98 ± 4.94 mmol/L) was much lower than that in survived patients (36.59 ± 4.85 mmol/L).

The creatinine was significantly different (*P* < 0.001) as the creatinine in dead patients (564.64 ± 268.80 *μ*moI/L) was much lower than that in survived patients (684.77 ± 271.00 *μ*moI/L).

### 3.3. Risk Factors for Death in Patients Receiving Peritoneal Dialysis Treatment

Based on the results of the comparison between survived patients and dead patients, we further analyzed the risk factors for death in patients receiving peritoneal dialysis treatment. As shown in Table 3, albumin, FBG, and creatinine were found to be significantly different.

However, the HR of creatinine was 0.999, with 95% CI of 0.998–1.000. Therefore, low albumin (HR = 2.254; 95% CI: 1.534–3.311; *P* < 0.001) and high FBG (HR = 1.474; 95% CI: 1.025–2.120; *P*=0.037) were considered to be risk factors.

### 3.4. Prognosis Prediction in Patients Receiving Peritoneal Dialysis Treatment

To evaluate the prognosis prediction value of the observed risk factors, ROC curves were drawn (Figure 1). FBG did not show the prediction value (*P*=0.593). Albumin (*P* < 0.001) and creatinine (*P* < 0.001) exhibited a value of prognosis prediction (Table 4). Of note, the albumin (with AUC of 0.683) showed a higher prognosis prediction value than creatinine (with AUC of 0.625).

The article "Low Serum Albumin Is Associated with Poor Prognosis in Patients Receiving Peritoneal Dialysis Treatment" was retracted in 2023. Reasons: signs of a paper mill; suspected computer-generated content; unreliable results or conclusions; concerns about the data.

### 3.5. Low Albumin and High FBG Were Associated with Poor Prognosis

Finally, the survival of patients receiving peritoneal dialysis treatment was analyzed (Figure 2). Both high FBG (*P*=0.005) and low albumin (*P* < 0.001) were associated with poor prognosis, and low albumin predicted a poorer survival.

## 4. Discussion

In this study, we found age, albumin, and creatinine were significantly different between dead and survived patients receiving peritoneal dialysis treatment. Albumin and creatinine showed the value of prognosis prediction. Furthermore, low albumin and high fasting blood glucose were risk factors and associated with poor prognosis. Thus, it is suggested that low albumin has a potential in predicting the prognosis of patients receiving peritoneal dialysis treatment.

To some extent, the level of albumin represents nutrition status and infection [11, 12]. Renal handling of albumin can influence renal function by the effects of albumin. Albumin filtration in glomeruli and tubular reabsorption are two major processes in the renal handling of albumin. The dysfunction of them leads to an increased excretion of albumin. Recently, Yamada et al. found lower serum albumin level is associated with an increased risk for loss of residual kidney function in patients receiving peritoneal dialysis treatment [13]. The loss of residual kidney function can make the general condition of patients worse and finally lead to the death. Our study goes further in exploring the prognosis prediction value of albumin by involving and considering the survival. Chiu et al. also reported lower serum albumin was associated with poorer survival [14]. Hao et al. used time-averaged albumin level and serum albumin reach rate as predictor variables and found higher serum albumin was associated with a lower all-cause mortality rate in patients undergoing long-term peritoneal dialysis treatment [15]. It is indicated that low serum albumin was a risk factor of both early and late death in incident peritoneal dialysis patients [16]. Interestingly, Singh et al. concluded that peritoneal dialysis is associated with lower mortality than hemodialysis in patients with low serum albumin [17]. As for the study of serum creatinine, Inaquma et al. reported the ratio of blood urea nitrogen to serum creatinine is associated with mortality by conducting a multicenter prospective cohort study [18].

By comparison of the age between dead and survived patients receiving peritoneal dialysis treatment, we found the age may influence the clinical outcomes and mortality. Consistent with the study conducted by Sakaci et al., mortality was higher in elderly patients and low albumin levels affected mortality [19]. The treatment of peritoneal dialysis should be cautious and based on accurate assessment, because of a higher incidence of intestinal complications, previous history abdominal surgeries, multiple comorbidities, and other possible contraindications [20, 21]. Our result also revealed that high fasting blood glucose may be associated with poor prognosis. Chen et al. reported the association of impaired fasting glucose and mortality in nondiabetic patients on maintenance peritoneal dialysis [22]. The role of high blood glucose in cardiovascular complications and even mortality of peritoneal dialysis treatment needs to be studied.

The article "Low Serum Albumin Is Associated with Poor Prognosis in Patients Receiving Peritoneal Dialysis Treatment" was retracted in 2023. Reasons: signs of a paper mill; suspected computer-generated content; unreliable results or conclusions; concerns about the data.

A number of researchers focus on the study of risk factors for mortality in patients receiving peritoneal dialysis treatment. Female gender, lower Kt/V (weekly urea clearance), and WCCr (weekly creatinine clearance) were found to be risk factors [23]. Lower hemoglobin levels and the presence of diabetes were shown to be risk factors as well [16].

In this study, common laboratory test indicators were analyzed to predict the prognosis of patients with peritoneal dialysis, which is helpful to advance treatment intervention for patients with possible poor prognosis and improve the prognosis of these patients. For patients with hypoalbuminemia and/or high FBG, which may lead to poor prognosis, dietary modification, intravenous albumin supplementation, and more stringent measures of blood glucose control may be considered. However, further prospective studies are needed to confirm the clinical efficacy of these measures.

This is a retrospective study, which is the major limitation. In the future study, we plan to involve the complications and causes of death. It is known that peritonitis has a notable association with peritoneal dialysis treatment since technique failure of peritoneal dialysis treatment could lead to peritonitis [24, 25]. The cardiovascular complication is another severe risk for peritoneal dialysis treatment [26]. The association of albumin and complication of peritoneal dialysis treatment is not clear and remains to be further studied.

### 4.1. Implications

Low albumin and high fasting blood glucose were risk factors and associated with poor prognosis. Low albumin has a potential in predicting the prognosis of patients receiving peritoneal dialysis treatment.

## Figures and Tables

**Figure 1:** ROC curve of albumin (a), creatinine (b), and FBG (c) for death risks in patients receiving peritoneal dialysis treatment.

**Figure 2:** (a) Survival of patients with high FBG (green line) and low and normal FBG (blue line). (b) Survival of patients with low albumin (green line) and high and normal FBG (blue line).

The article "Low Serum Albumin Is Associated with Poor Prognosis in Patients Receiving Peritoneal Dialysis Treatment" was retracted in 2023. Reasons: signs of a paper mill; suspected computer-generated content; unreliable results or conclusions; concerns about the data.

**Table 1:** Characteristics of patients receiving peritoneal dialysis treatment.

Characters	Mean (median)	SD (quartile spacing)	*n*
Age	62.51	14.07	301
Male	—	—	147
Female	—	—	178
Survival time (d)	892.36	716.22	325
Systolic pressure (mmHg)	143.46	48.71	325
Diastolic pressure (mmHg)	80.81	14.73	325
Pulse (beat per minute)	77.83	11.60	313
Total protein (g/L)	65.54	25.18	323
Albumin (g/L)	34.89	5.20	323
Ca^2+^ (mmol/L)	2.21	0.28	323
Phosphate (mmol/L)	1.38	0.52	318
K^+^ (mmol/L)	4.19	0.89	324
Na^+^ (mmol/L)	139.79	2.93	323
Cl^−^ (mmol/L)	99.39	9.90	322
Fasting blood glucose (mmol/L)	7.63	3.92	323
Blood urea nitrogen (mmol/L)	19.68	32.59	323
Creatinine (*μ*moI/L)	628.24	276.15	323
Hemoglobin (g/L)	114.04	(101–129)	325
Parathyroid hormone (pg/mL)	146.90	(55.46–270.90)	325

**Table 2:** Comparisons between survival and death.

	Survival (*n* = 173)	Death (*n* = 152)	*t* (*x*^2^)	*P* value
Age	28.75 ± 13.13	66.96 ± 13.89	5.267	<0.001
Male	78	67	0.859	0.651
Female	93	85		
Survival time (d)	965.59 ± 794.95	809.02 ± 606.39	1.975	0.049
Systolic pressure (mmHg)	146.72 ± 63.41	139.74 ± 22.05	1.289	0.198
Diastolic pressure (mmHg)	82.32 ± 16.01	79.08 ± 12.96	1.990	0.047
Pulse (beat per minute)	77.63 ± 11.21	78.05 ± 12.05	0.325	0.745
Total protein (g/L)	67.77 ± 33.77	63.04 ± 7.49	1.688	0.092
Albumin (g/L)	36.59 ± 4.85	32.98 ± 4.94	6.621	<0.001
Ca^2+^ (mmol/L)	2.22 ± 0.29	2.20 ± 0.26	0.624	0.533
Phosphate (mmol/L)	1.40 ± 0.51	1.36 ± 0.53	0.729	0.467
K^+^ (mmol/L)	4.29 ± 0.84	4.09 ± 0.95	2.035	0.322
Na^+^ (mmol/L)	139.97 ± 2.95	139.60 ± 2.91	1.128	0.260
Cl^−^ (mmol/L)	99.84 ± 9.24	98.89 ± 10.60	0.861	0.390
FBG (mmol/L)	7.43 ± 3.87	7.86 ± 3.97	0.970	0.333
BUN (mmol/L)	21.65 ± 44.15	17.47 ± 7.75	1.151	0.251
Creatinine (*μ*moI/L)	684.77 ± 271.00	564.64 ± 268.80	3.992	<0.001
Hemoglobin (g/L)	117.54 ± 23.72	112.19 ± 22.25	2.085	0.038
PTH (pg/mL)	212.30 ± 203.37	208.34 ± 275.71	0.148	0.882

*Note.* FBG: fasting blood glucose; BUN: blood urea nitrogen; PTH: parathyroid hormone.

**Table 3:** Risk factors for death in patients receiving peritoneal dialysis treatment.

		*P* value	HR	95% CI	
				Lower	Upper
PTH	75–150	0.410	1.000	—	—
	<75	0.110	1.481	0.915	2.398
	150–300	0.618	1.136	0.688	1.877
	>300	0.335	1.282	0.774	2.126

Albumin	Normal		1.000	—	—
	Low	<0.001	2.254	1.534	3.311

Cl^−^	Normal	0.853	1.000	—	—
	Low	0.971	1.010	0.586	1.740
	High	0.574	1.201	0.634	2.275

Na^+^	Normal	0.357	1.000	—	—
	Low	0.947	0.974	0.442	2.143
	High	0.152	0.230	0.031	1.716

K^+^	Normal	0.423	1.000	—	—
	Low	0.314	1.246	0.812	1.911
	High	0.433		0.335	1.598

Phosphate	Normal	0.313	1.000	—	—
	Low	0.747	1.075	0.692	1.671
	High	0.129	1.453	0.897	2.354

Ca^2+^	Normal	0.347	1.000	—	—
	Low	0.788	0.946	0.629	1.422
	High	0.147	0.411	0.123	1.367

Hypertension	No		1.000	—	—
	Yes	0.789	1.048	0.741	1.483

Hemoglobin	Normal	0.386	1.000	—	—
	Low	0.531	0.841	0.489	1.445
	High	0.272	0.430	0.095	1.939

FBG	Normal	0.112	1.000	—	—
	Low	0.680	1.220	0.474	3.137
	High	0.037	1.474	1.025	2.120

Sex	Male		1	—	—
	Female	0.515	0.881	0.601	1.290

Age		0.102	0.966	0.978	1.002

Creatinine		0.022	0.999	0.998	1.000

*Note.* FBG: fasting blood glucose; PTH: parathyroid hormone.

The article "Low Serum Albumin Is Associated with Poor Prognosis in Patients Receiving Peritoneal Dialysis Treatment" was retracted in 2023. Reasons: signs of a paper mill; suspected computer-generated content; unreliable results or conclusions; concerns about the data.

**Table 4:** ROC curve in patients receiving peritoneal dialysis treatment.

Predictors	ROC curves			
	Cut-off value	AUC	95% CI	p value
Albumin	35.75	0.683	0.626–0.739	<0.001
Creatinine	711.50	0.625	0.565–0.684	<0.001
Fasting blood glucose	4.44	0.483	0.422–0.545	0.593

## Data Availability

The data used to support the findings of this study are included within the article.
